RETRACTED

# Research on the efficacy of *Celastrus Orbiculatus* in suppressing TGF-β1-induced epithelial-mesenchymal transition by inhibiting HSP27 and TNF-α-induced NF-κB/Snail signaling pathway in human gastric adenocarcinoma

**DOI:** 10.1186/1472-6882-14-433

**Published:** 2014-11-05

**Authors:** Yaodong Zhu, Yanqing Liu, Yayun Qian, Xiaojun Dai, Ling Yang, Jue Chen, Shiyu Guo, Tadashi Hisamitsu

**Affiliations:** Institute of Combining Chinese Traditional and Western Medicine, Medical College, Yangzhou University, Yangzhou, Jiangsu 225001 China; Jiangsu Key Laboratory of Integrated Traditional Chinese and Western Medicine for Prevention and Treatment of Senile Disease, Yangzhou, Jiangsu 225001 China; Department of Physiology, School of Medicine, Showa University, Tokyo, 142 Japan

**Keywords:** *Celastrus orbiculatus*, Gastric cancer, Epithelial-mesenchymal transition, HSP27, NF-κB

## Abstract

**Background:**

*Celastrus orbiculatus* has been used as a folk medicine in China for the treatment of many diseases. In the laboratory, the ethyl acetate extract of *Celastrus orbiculatus* (COE) displays a wide range of anticancer functions. However, the inhibition of the metastasis mechanism of COE in gastric cancer cells has not been investigated so far.

**Methods:**

The present study was undertaken to determine if the anti-metastasis effect of COE was involved in inhibiting of epithelial–mesenchymal transition (EMT) of human gastric adenocarcinoma SGC-7901 cells. *In vitro*, a well-established experimental EMT model involving transforming growth factor β1 (TGF-β1) was applied. Viability, invasion and migration, protein and mRNA expression of tumor cells were analyzed by MTT assay, transwell assay, western blot and real-time PCR, respectively. The molecular targets of COE in SGC-7901 cells were investigated by two-dimensional gel electrophoresis (2-DE) and MALDI-TOF-TOF mass spectrometer. Overexpression of heat shock protein 27 (HSP27) was performed by transfected with the recombinant retroviral expression plasmid. *In vivo*, the anti-metastasis mechanisms of COE in the peritoneal gastric cancer xenograft model was explored and the effect was tested.

**Results:**

The non-cytostatic concentrations of COE effectively inhibited TGF-β1 induced EMT process in SGC-7901 cells, which is characterized by prevented morphological changes, increased E-cadherin expression and decreased Vimentin, N-cadherin expression. Moreover, COE inhibited invasion and migration induced by TGF-β1. Using a comparative proteomics approach, four proteins were identified as differently expressed, with HSP27 protein being one of the most significantly down-regulated proteins induced by COE. Moreover, the activation of nuclear factor κB (NF-κB)/Snail signaling pathway induced by tumor necrosis factor-α (TNF-α) was also attenuated under the pretreatment of COE. Interestingly, overexpression of HSP27 significantly decreases the inhibitory effect of COE on EMT and the NF-κB/Snail pathway. Furthermore, COE significantly reduced the number of peritoneal metastatic nodules in the peritoneal gastric cancer xenograft model.

RETRACTED

**Conclusions:**

Taken together, these results suggest that COE inhibits the EMT by suppressing the expression of HSP27, correlating with inhibition of NF-κB/Snail signal pathways in SGC-7901 cells. Based on these results, COE may be considered a novel anti-cancer agent for the treatment of metastasis in gastric cancer.

## Background

Gastric cancer is the most common gastrointestinal cancer originating from the epithelium and is a serious threat to human health. Most patients are diagnosed at an advanced stage, with metastasis and poor prognosis [1]. Metastasis of gastric cancer is not only a sign of deterioration, but also the major cause of treatment failure and death [2]. Therefore, effective therapeutic agent targeting the cancer metastasis is significant for gastric cancer treatment. Epithelial-mesenchymal transition (EMT), the process of cells losing their epithelial phenotype and acquiring a migratory mesenchymal phenotype, has been accepted to play an important role in cancer metastasis in several human malignancies including gastric cancer [3]. Thus, EMT could be a very promising therapeutic target, and the inhibition of EMT may prevent or restrain the metastasis of gastric cancer [4].

Increasing evidence suggests that some Chinese herbal medicine, containing some bioactive compounds or a variety of phytochemicals, may inhibit EMT and reduce metastasis [5–7]. Thus, some herbs can be utilized as complementary and alternative treatments and as adjuvant therapy for conventional cytotoxic therapies. *Celastrus orbiculatus* (Celastraceae), has been used as a folk medicine in China for the treatment of many diseases, including arthritis and other inflammatory diseases. It was found that the ethyl acetate extract of *Celastrus orbiculatus* (COE) displays anti-cancer effects *in vitro* and *in vivo* through the inhibition of proliferation, angiogenesis, invasion and metastasis ability [8, 9]. Although COE has been reported in various bioactivity assays, the molecular mechanism by which it modulates the EMT-mediated alteration of human gastric cancer cells has not been elucidated so far.

In this study, we investigated the effects of COE on transforming growth factor β1 (TGF-β1) induced EMT *in vitro* and tumor metastasis *in vivo* and explored the underlying molecular mechanism. The results indicated that COE inhibited the EMT and tumor metastasis by suppressing the expression of HSP27, correlating with inhibition of NF-κB/Snail signal pathway in SGC-7901 cells. Therefore, the present findings suggest that COE might have potential therapeutic effect against gastric cancer.

RETRACTED

## Methods

### Reagents and antibodies

RPMI-1640 and fetal bovine serum (FBS) was acquired from Gibco-BRL (Gaithersburg, MD, USA). 3-(4,5-dimethyl-2-thiazyl)-2,5-diphenyl-2H-tetrazolium bromide (MTT) was purchased from Sigma Chemical Co. (St. Louis, MO, USA). Recombinant TGF-β1 and TNF-α were obtained from R&D systems (Minneapolis, MN, USA). Matrigel was purchased from BD Biosciences (San Jose, CA, USA). Antibodies against E-cadherin, N-cadherin, Vimentin, HSP27, Snail, NF-κB p65, IκBα, phosphorylation of IκBα, Histone H3 and β-actin were purchased from Cell Signaling Technology (Beverly, MA, USA). Other chemicals used were of analytical grade from commercial sources.

### Plant material and extraction

The plant materials were purchased from Guangzhou Zhixin Pharmaceutical Co. Ltd. (Guangzhou, China) in 2007. The COE was prepared at the department of Chinese Materia Medica Analysis, China Pharmaceutical University (Nanjing, China). The preparation procedure has been described previously [10]. Briefly, dried stems of *Celastrus orbiculatus* were minced, extracted with 95% ethanol, filtered, and evaporated to dryness. The extract was evacuated with a membrane pump to remove residual solvent. The aqueous layer was then partitioned from the ethanol extract with ethyl acetate. Finally, the ethyl acetate extract was condensed and lyophilized into powder and stored at 4°C. The chemical constituents from the stems of *Celastrus orbiculatus* were investigated and compounds were isolated as previously described. 23-hydroxybetulonic acid, 23-hydroxy-3-oxoolean-12-en-28-oic acid, oleanolic acid, 3-oxo-24-norolean-12-en-28-oic acid and wilforlide B were confirmed to be included in the extract by High Performance Liquid Chromatography (HPLC) assay [11, 12]. The resultant COE micropowder was dissolved in dimethyl sulfoxide (DMSO; Sigma, St Louis, MO, USA) and diluted to different concentrations before use.

### Cell culture

The human gastric adenocarcinoma cell line SGC-7901 was obtained from the Cell Bank of Chinese Academy of Sciences Shanghai Institute of Cell Biology (Shanghai, China). SGC-7901 cells were cultured in RPMI1640 containing 10% FBS and maintained at 37°C in a humidified incubator in an atmosphere of 5% CO_2_.

### Cell viability assay

The cell viability was measured using the MTT assay. SGC-7901 cells were seeded in a 96-well plate and treated with COE at various concentrations (20, 40, 80,160 and 320 μg/mL) in triplicate. After 24 h incubation, cell viability was determined by being incubated with medium containing MTT for 4 h, followed by dissolving the formazan crystals with DMSO. The absorbance at 490 nm was determined by a microplate reader and presented as relative cell viability. The tests were performed at least three independent times.

RETRACTED

### Cell invasion and migration assays

According to manufacturer’s instruction, cell invasion and migration assays were performed using a transwell membrane (Corning Costar Corporation, Cambridge, MA, USA). In the invasion assay, Matrigel was applied to the upper chamber. Cells were seeded into the upper chamber and treated with different concentrations of COE. Medium containing 10% FBS and TGF-β1 were added to the lower chamber for 24 h as a chemoattractant. At the end of the treatment, the cells on the upper surface of the membrane were removed by cotton swabs and cells invaded across the Matrigel to the lower surface of the membrane were fixed with methanol and stained with crystal violet. Images were obtained under a microscope at × 200 magnification (Nikon, Chiyoda-Ku, Tokyo, Japan) and invading cells were quantified by manual counting. Migration assays were carried out in the same procedure, except that the polycarbonate membrane was not coated with matrigel. Each experiment was repeated three times.

### Two-dimensional gel electrophoresis and image analysis

Two-dimensional gel electrophoresis (2-DE) was performed as previously reported [13]. Briefly, protein samples (2 mg), extracted from untreated controls, TGF-β1 treated cells, and COE-treated cells were subjected to isoelectric focusing using the PROTEAN IEF Cell System (Bio-Rad, USA). For the second dimension, focused samples in the strips were subjected to electrophoresis using a PROTEAN II xi system (Bio-Rad). The gels were then stained with Coomassie Brilliant Blue (CBB) to assign the protein pI and MW, respectively. Image acquisition and analysis were performed with GS-800 Calibrated Densitometer (Bio-Rad) and PDQuestâ„¢ 2-DE Analysis Software (Bio-Rad). The protein expression level was determined of using the relative volume of each spot in the gel. Protein spots with more than 2-fold significant change in density in a consistently increased or decreased direction were considered to be differentially expressed, and were selected for further identification.

### Mass spectrometry and database searching

The protein spots were used for identification by MALDI-TOF/TOF using an ABI 5800 Proteomics Analyzer with delayed ion extraction (Applied Biosystems, USA). The database search was performed by using the MASCOT search engine (Matrix Science, London, United Kingdom) to screen the NCBI protein sequence database restricted to human taxonomy. All the identified proteins should have a protein score more than 64 and individual ion score more than 30.

RETRACTED

### Western blot analysis

Nuclear and cytosolic fractions were prepared by using Nuclear and Cytoplasmic Extraction Reagents kit (Fermentas, Canada). Histone H3 and β-actin were used as markers for nuclear and cytosol proteins, respectively. Lysate proteins were resolved by SDS-PAGE and transferred into nitrocellulose membranes (Millipore, Bedford, MA, USA). The blot was blocked in blocking buffer (5% not-fat dry milk and 1% Tween-20 in PBS) for 2 h at room temperature, and then incubated with appropriate primary antibodies in blocking buffer overnight at 4°C. Subsequently, the membranes were washed and incubated with secondary antibodies for 2 h at room temperature. Enhanced chemiluminescence was used to detect a signal using the SuperSignal West Pico Chemiluminescent Substrate (Thermo Scientific, Rockford, USA) on a Molecular Imager ChemiDoc XRS System (Bio-Rad). Densitometry was determined using Quantity One Analysis Software (Bio-Rad).

### Quantitative real-time PCR (qRT-PCR)

Total RNA was extracted from the cells using the Trizol reagent (Invitrogen, Carlsbad, USA) and exactly following the instruction of manufacturer’s manual under RNase-free condition. After complementary DNA was synthesized with a two-step reverse transcription reaction kit (TaKaRa, Dalian, China), qRT-PCR was performed on an Applied Biosystems 7500 Real-time PCR System using SYBR Premix Ex Taq Kit (TaKaRa) in Axygen 96-well reaction plates following the manufacturer’s protocols. Primers were obtained from Shanghai Sangon Biological Engineering Technology and Services (Shanghai, China) and their sequences were:

HSP27 (NM_001540.3), forward primer 5′-AGT GGT CGC AGT GGT TAG-3′, reverse primer 5′-CAG GGA GGA GGA AAC TTG-3′; GAPDH (NM_002046), forward primer 5′-TGG CAC CCA GCA CAA TGA A-3′, reverse primer 5′-CTA AGT CAT AGT CCG CCT AGA-3′. The level of GAPDH mRNA transcript was used to normalize all reported gene expression levels, and the data were analyzed using the 2^-ΔΔCt^ method.

### Transfection and luciferase reporter gene assay

Briefly, SGC-7901 cells at 1 × 10^6^ cells per well were plated in 6-well plates and grown to approximately 70% confluence. Then, the cells were transiently co-transfected with pGL6-NF-κB-TA-luc (Beyotime Institute Biotechnology, China) and pRL-TK (Promega, USA) for normalizing transfection efficacy. Six hours after transfection, the cells were incubated with COE for 1 h followed by TNF-α (10 ng/mL) activation for 24 h. The cells were harvested in lysis buffer (Promega) and were assayed by using the dual luciferase system (Promega). The results were normalized to the luciferase activity of the internal control.

RETRACTED

### Retrovial constructs and transfection

The whole codon sequence of HSP27 (NM_001540.3) was PCR amplified using Platinums Taq DNA Polymerase high fidelity (Invitrogen, Carlsbad, CA, USA) and primers: forward 5′-ATA GAT CTA TGA CCG AGC GCC GCC GCG TCC CCT TC -3′, reverse 5′-AGC TCG AGT TAC TTG GCG GCA GTC TCA-3′. The PCR product was cloned into Bgl II and XhoI of retroviral vector MSCV MIGR1 (kindly provided by professor Yu D from University of Pennsylvania). Sequence fidelity was confirmed by DNA sequencing. SGC-7901 cells were seeded in 6-well plates (2 × 10^5^ cells/well) overnight and transfected with the recombinant retroviral expression plasmid using Lipofectamine 2000 (Invitrogen) according to the manufacturer’s instructions. The cells were visualized under a fluorescence microscope (Nikon, Chiyoda-Ku, Tokyo, Japan) to detect transfection efficiency and treated with COE for another 24 h.

### Animal studies

Male athymic nude BALB/c mice were obtained from the Comparative Medicine Laboratory Animal Center [License No. scxk (SU) 2012-0004] of Yangzhou University (Jiangsu, China). The mice aged 6 weeks were maintained under specific pathogen-free conditions. The experiments were carried out in accordance with internationally accepted guidelines on the use of laboratory animals, and the protocols were approved by the Institutional Animal Care and Use Committee (IACUC) of Yangzhou University. To generate the intraperitoneal xenograft model, SGC-7901 cells (1 × 10^7^ per mouse) were suspended in 100 μL of PBS, and injected on day 0 into the abdominal cavity. The mice were randomly divided into blank control group, negative control group (1% DMSO), positive control group (xeloda), and low-dose, medium-dose and high-dose COE groups (10, 20 and 40 mg/kg, respectively).

Treatment started 2 weeks after the SGC-7901 cells were injected and continued for 3 weeks. The growth of the mice was monitored regularly. After 3 weeks of treatment, all the mice were dead and laparotomy was performed. Peritoneal nodules that had grown to a diameter above 1.0 mm were counted. Body-weight changes was also monitored.

### Statistical analysis

The results are expressed as the means±SD. Each experiment was repeated at least three times. Applying Student’s t-test, the differentiation of Statistical analysis of two samples was performed. Statistical comparisons of more than two groups were performed using one-way analysis of variance (ANOVA) with Bonferroni’s post hoc test. All statistical analysis were performed using SPSS for Windows, version 10 (SPSS, Inc.). *P* values below 0.05 were considered statistically significant.

RETRACTED

## Results

### COE inhibits TGF-β1-induced EMT in SGC-7901 cells

First, the effect of COE on cell viability with the MTT assay was examined at 24 h. As shown in Figure 1A, COE inhibited the viability of SGC-7901 cells in a concentration-dependent manner. The data indicated that less than 20 μg/mL COE had no influence on cell viability, while 40 μg/mL COE significantly inhibited SGC-7901 cell viability. The non-cytostatic concentrations (below 20 μg/mL) of COE was chosen for further experiments to guarantee that inhibition of COE for TGF-β1-induced EMT was not due to inhibition of proliferation.

To more fully investigate the effect of COE on TGF-β1 stimulated EMT process, SGC-7901 cells were incubated with or without COE (5, 10 and 20 μg/mL) for 1 h followed by treatment with 10 ng/mL TGF-β1 for 24 h. Then cells were examined and photographed under a phase-contrast microscope. As shown in Figure 1B, treatment with TGF-β1 induced prominent morphological changes in SGC-7901 cells, including elongated and spindle-like shapes, which were noticeably suppressed by pretreatment with COE. Meanwhile, TGF-β1 induced cell invasion and migration were inhibited by COE in a concentration-dependent manner (Figure 1C). To further confirm the effects of COE on TGF-β1-induced EMT, we examined the effect of COE on expression of EMT markers by western blot assay. The results showed that addition of 10 ng/mL TGF-β1 reduced E-cadherin expression while it increased Vimentin and N-cadherin expression. Interestingly, pretreatment with COE effectively prevented these expressional variations in a concentration-dependent manner (Figure 1D). These findings showed that COE inhibited the effects of TGF-β1 induced EMT in SGC-7901 cells.

**Figure 1:** **COE inhibits TGF-β1 induced EMT in SGC-7901 cells. (A)** The effect of COE on the viability of SGC-7901 cells, as measured with the MTT assay. SGC-7901 cells were either untreated or treated with 20, 40, 80, 160, 320 μg/mL of COE for 24 h. Results are presented as means±SD of three assays. **P <0.01, compared with the untreated control. **(B)** Morphological changed between TGF-β1-treated SGC-7901 cells and TGF-β1-treated SGC-7901 cells with COE. SGC-7901 cells were incubated with COE (5, 10, 20 μg/mL) for 1 h followed by treatment with 10 ng/mL TGF-β1 for 24 h. Representative pictures of cells treated with COE showed that epithelial morphology of cells was maintained even in the presence of TGF-β1 (200 × magnification). **(C)** The effect of COE on TGF-β1-induced invasion and migration in SGC-7901 cells were assessed using transwell assay. The invasion and migration ability of cells were quantified by counting the number of cells that invaded to the underside of the porous polycarbonate membrane under microscope (200 × magnification). **(D)** The effect of COE on the expression of EMT markers. The expression of epithelial marker, E-cadherin and mesenchymal markers, N-cadherin, Vimentin were evaluated by western blot. β-actin was served as an internal control of protein level. The relative density of EMT markers was normalized to β-actin, which was determined by densitometric analysis. Values are expressed as means±SD of three independent experiments. #*P* <0.05, ##*P* <0.01, compared with control. *P <0.05, **P <0.01, compared to TGF-β1-treated cells.

RETRACTED

### Proteomics analysis

To explore the target-specific proteins of COE inhibits TGF-β1 induced EMT, differential protein expression of control, TGF-β1, and COE treated groups using 2-DE based proteomics were monitored. Proteins were separated in the 2-D gels in the ranges of MW 14-100 kDa and pI 3-10. Overall, approximately 500 spots were detected on each gel and 80% were matched between gels (Figure 2A). Image analysis revealed that a number of protein spots were significantly altered in terms of volume intensity. Prominent areas in arrows are the locations where protein alterations were detected. There were four protein spots which were promoted in TGF-β1 treated group compared with control group, but depressed in the COE treated group. These differentially expressed spots were successfully identified by MALDI-TOF/TOF and MS/MS analysis. The characteristics of all identified proteins, including protein name, NCBI accession number, molecular mass/pI, protein score and coverage were all summarized in Table 1. In addition, the representative MS map for the protein identification was shown in Figure 2B. Our data suggest that COE maybe plays an anti-EMT effects through comprehensively regulating the functional proteins such as HSP27, prohibitin, cofilin-1, and Annexin A5, et al.

**Figure 2:** **Differential protein expression profiles of control, TGF-β1, and COE treated SGC-7901 cell samples. (A)** Approximately 2 mg of protein lysates were focused on pH 3-10 linear IPG strips and then separated by a 12% polyacrylamide gel. Protein expression patterns were subsequently visualized by Coomassie Brilliant Blue staining method. Spots highlighted in arrows were the areas where significant and consistent differences were expressed in the protein expression levels in control, TGF-β1, and COE treated groups. **(B)** Identification and verification of candidate proteins by MALDI-MS analyses. The mass spectrometric spectra showed the identities of the proteins, namely (i) HSP 27, (ii) prohibitin, (iii) cofilin-1, and (iv) Annexin A5.

RETRACTED

**Table 1:** **List of identified proteins in proteomic study**

Spot	Protein	Accession no.	Theoretical Mw (Da) /pI	Score	Sequence coverage
1	Heat shock protein 27	gil662841	22427/7.83	212	31%
2	Prohibitin	gil4505773	29843/5.57	633	40%
3	Cofilin-1	gil5031635	18719/8.22	517	53%
4	Annexin A5	gil809185	35840/4.94	406	37%

### COE modifies the endogenous level of HSP27 and inhibits TNF-α-induced activation of NF-κB/Snail in SGC-7901 cells

Previous studies had shown that HSP27 was a critical mediator in cancer progression [14]. In the proteomics analysis, it was found that the most dramatically altered protein was HSP27 (3.2-fold down-regulation). Therefore, this protein was paid particular attention in the research. Dose-dependent down-regulation of HSP27 after COE treatment was confirmed by western blot analysis in SGC-7901 cells (Figure 3A). To get a hint how COE affects HSP27, qRT-PCR was used to detect the HSP27 mRNA level. As shown in Figure 3B, HSP27 mRNA level was not significantly altered after treated with COE, while the level of HSP27 protein was reduced. These results showed that COE could decrease the HSP27 protein level without modulating the expression of its mRNA transcripts levels. In order to measure effects of COE on degradation of HSP27 protein, cells were treated with the proteasome inhibitor MG132. And we found that MG132 upregulated the level of HSP27 induced by TGF-β1 when treated with COE (Figure 3C). This suggests that an increased degradation of HSP27 occured in SGC-7901 cells treated with COE. Taken together our results indicate that HSP27 played a critical role in COE-inhibited EMT.

**Figure 3:** **COE modifies the endogenous level of HSP27 and inhibits TNF-α-induced activation of NF-κB/Snail in SGC-7901 cells. (A)** COE suppresses TGF-β1 induced HSP27 expression. SGC-7901 cells were treated with TGF-β1 (10 ng/mL) or with TGF-β1 and COE (5, 10, 20 μg/mL) for 24 h. The expression levels of HSP27 was analyzed by western blot assay. **(B)** The level of HSP27mRNA was examined by qRT-PCR using total mRNA of SGC-7901 cells and compared with TGF-β1 alone. The data was analyzed using the 2^-ΔΔCt^ method. **(C)** Cells were treated with COE and/or TGF-β1 (10 ng/mL) in the presence or absence of the proteasome inhibitor MG132 (1 μM). HSP27 content was evaluated by western blot. **(D)** Effect of COE on TNF-α-mediated activation of NF-κB/Snail signal pathway. Cells were pretreated with COE (5, 10, 20 μg/mL) for 1 h, and then TNF-α (10 ng/mL) was added for another 6 or 12 h. Nuclear and cytoplasmic fractions were separated by a nuclear extract kit, and the expression levels of the NF-κB p65, Snail, IκBα and phosphorylation of IκBα protein were measured by western blot analysis. **(E)** Effect of COE on TNF-α-induced activation of NF-κB. SGC-7901 cells were transiently co-transfected with pGL6-NF-κB-TA-luc and pRL-TK. After 6 h, the cells were incubated with COE for 1 h followed by TNF-α (10 ng/mL) activation for 24 h. The transcriptional activity of NF-κB was determined by luciferase reporter gene assay and normalized to the internal control. The results are representative of at least three independent experiments. #*P* <0.05, ##*P* <0.01, compared with control. *P <0.05, **P <0.01, compared to TGF-β1 or TNF-α-treated cells.

RETRACTED

It was also reported that HSP27 maintains a population of breast cancer stem cells that display EMT characteristics by increasing degradation of IκBα, enhancing nuclear translocation of NF-κΒ and stabilizing Snail [15]. On the basis of these facts, it was hypothesized that COE could inhibit EMT by modulating HSP27 and NF-κB/Snail signal pathway. Therefore, we proceeded to explore whether the anti-EMT effect of COE is associated with the inhibition of NF-κB/Snail activation. Our results demonstrated that TNF-α (classic NF-κB pathway activator) promoted the expression of NF-κB p65, phosphorylation of IκBα, and Snail protein, accompanied by a decreased expression of IκBα, and this effect was abrogated by COE (Figure 3D). Besides, the research also showed that the enhancement of NF-κB transcriptional activity by TNF-α was also inhibited by COE using an NF-κB mediated luciferase reporter gene assay (Figure 3E). This results support previous hypothesis that COE might inhibit EMT via the regulation of the NF-κB/Snail pathway.

### The role of HSP27 in COE-mediates inhibition of EMT and NF-κB/Snail signal pathway

To confirm the role of HSP27 in COE inhibits EMT in SGC-7901 cells, the recombinant retrovirus plasmid MIGR1-HSP27 containing full length of human HSP27 gene was successful constructed. The constructed plasmid MIGR1-HSP27, empty plasmid MIGR1 were transfected into SGC-7901 cells and the cells were selected by flow cytometry for GFP + cells, a transduction efficiency of close to 100% was achieved (Figure 4A). Western blot analysis indicated that HSP27 overexpression by recombinant retrovirus plasmid transfections in SGC-7901 cells not only increased HSP27 content but also reproduced EMT features classically induced by TGF-β1 (Figure 4B). Subsequently, the overexpression HSP27 cell line and control cell line were pretreated with or without COE (20 μg/mL) for 1 h and then stimulated with 10 ng/mL TGF-β1 for 24 h. As shown in Figure 4C, COE treatment caused suppression of HSP27 level in control cells as well as in HSP27 overexpressed cells. The effects of COE on the upregulation of E-cadherin and downregulation of N-cadherin and Vimentin were also blocked by HSP27 overexpression. In addition, HSP27 overexpression blocked the effects of COE on cell invasion and migration (Figure 4D). More importantly, we sought to determine whether HSP27 is involoved in the COE-mediated inhibition of NF-κB/Snail signal pathway. As shown in Figure 4E, the overexpression of HSP27 decreased the inhibitory effect of COE on the nuclear translocation of NF-κB p65 and Snail, as well as the phosphorylation of IκBα. These results indicated that HSP27 may play a critical role in COE inhibits EMT by inhibiting NF-κB/Snail signal pathway.

RETRACTED

**Figure 4:** **The role of HSP27 in COE-mediates inhibition of EMT and NF-κB/Snail signal pathway. (A)** Overexpression of HSP27 was performed by transfected with the recombinant retroviral expression plasmid and the cells were selected by flow cytometry for GFP + cells. Nearly 100% transduction efficiency was achieved as shown by fluorescent microscope. **(B)** Expression of HSP27, E-cadherin, N-cadherin, Vimentin were analyzed by western blot in SGC-7901 cells that were transfected with control (empty) or HSP27 vectors or treated with TGF-β1 (10 ng/mL). β-actin was served as an internal control of protein level. The relative density was normalized to β-actin, which was determined by densitometric analysis. Values are expressed as means±SD of three independent experiments. **P <0.01, compared with control. ##*P* <0.01, compared to MIGR1 group. **(C)** The overexpression HSP27 cell line and control cell line were treated with or without COE (20 μg/mL) for 1 h followed by TGF-β1 (10 ng/mL) for 24 h, and the protein expression of HSP27, E-cadherin, N-cadherin, Vimentin were detected by western blot analyses. β-actin was served as an internal control of protein level. **(D)** Cell invasion and migration were analyzed by transwell assay. The quantitative data was presented as means±SD of three independent experiments. **(E)** The overexpression HSP27 cell line and control cell line were treated with or without COE (20 μg/mL) for 1 h followed by TNF-α (10 ng/mL) for 24 h, and the protein expression of IκBα, p-IκBα, NF-κB p65 and Snail were detected by western blot analyses. β-actin and H3 were served as an internal control of protein level. **P <0.01 compared with the respective untreated control (MIGR1 or MIGR1-HSP27). ##*P* <0.01 compared COE-treated MIGR1 group compared with COE-treated MIGR1-HSP27 group.

RETRACTED

### COE blocked peritoneal metastasis of gastric cancer *in vivo*

The *in vitro* data prompted us to test the anti-metastasis activity of COE in mice harboring a intraperitoneal xenograft model of SGC-7901 cells. The results of our previous toxicity assessment experiments suggested that the *in vivo* dosage of COE should not exceed 40 mg/kg (data not shown). Therefore, 10, 20, and 40 mg/kg were used in these experiments. We examined whether COE resulted in inhibition of peritoneal dissemination, by counting the macroscopic nodules of peritoneal dissemination at the end of the experiment. As shown in Figure 5A, the gross findings in the mesentery of the control group were clearly different from those in the other groups. The number of metastatic nodules above 1 mm was significantly reduced in COE treated groups than that in the control group (Figure 5B). Moreover, the average body weight of the mice in the COE and control groups was not significantly different throughout the experiment (Figure 5C). These data indicated that there was little to no toxicity of COE at doses of 10, 20 and 40 mg/kg under the same treatment conditions. Western blot analyses were performed to detect the expression levels of HSP27 in the xenograft tumors. The results revealed a decrease in the expression of HSP27 in the COE treatment groups compared with the control group (Figure 5D).

**Figure 5:** ***In vivo*** **anti-metastasis effect of COE. (A)** Macroscopic appearance of peritoneal tumors was established by intraperitoneal inoculation of SGC-7901 cells. Arrows indicated peritoneal metastatic tumor in each group. Markedly fewer peritoneal metastases were found in mice in high-dose COE group (40 mg/kg) and positive control group (xeloda). **(B)** Number of peritoneal metastatic nodules (above 1 mm) in each group. High-dose COE group (40 mg/kg) and positive control group (xeloda) significantly suppressed the development of peritoneal metastases. **(C)** The average body weight of the mice in the COE groups did not decrease significantly throughout the experiment. **(D)** Western blot analyses confirmed decreased HSP27 expression in COE-treated tumors. β-actin was served as an internal control of protein level. All values are presented as the means±SD, *P <0.05, **P <0.01, as compared with the control group.

## Discussion

COE is the product isolated from the plant of *Celastrus orbiculatus*, a Chinese traditional herb. In recent years, a number of experimental studies on COE have been performed worldwide. COE has revealed distinct anti-tumor activity, such as the inhibition of cell proliferation, induction of cell apoptosis, inhibition of angiogenesis, and inhibition of invasion and metastasis [8, 9, 16, 17]. Although several reports have suggested that the function of COE are related with tumor metastasis, its role in EMT has not been examined.

RETRACTED

Many studies have reported that EMT has a potential mechanism for the metastasis of cancer cells [18]. EMT is a biological process in which epithelial cells undergo from phenotypic conversion to mesenchymal cells [19]. During EMT, the ability of an epithelial cell to change its morphological characteristics to a mesenchymal cell is a fundamental process in tumorigenesis [18]. The reduction of E-cadherin expression is a representative characteristic of EMT and is an important part of the metastatic process [20]. It demonstrated that COE suppressed TGF-β1-induced epithelial cell marker (E-cadherin) downregulation and mesenchymal cell marker (N-cadherin, Vimentin) upregulation while retaining epithelial morphology. Thus, our results indicate that COE treatment inhibits the TGF-β1 mediated EMT process and retains epithelial morphology in SGC-7901 cells.

Proteomic expression profiling is a powerful approach for the identification of potential molecular targets [21]. In the present study, four protein spots were successfully identified, the most dramatically altered protein was HSP27 (3.2-fold down-regulation). Therefore, we selected HSP27 for further study. Heat shock proteins (HSPs) are a group of molecular chaperons which are induced by a variety of physiological and environmental insults, playing important roles in regulating signaling and transcriptional survival networks to facilitate cells to survive to otherwise lethal conditions [22]. HSP27 is a major member of the small HSPs family and its over-expression is suggested to be correlated with tumorigenesis, chemo-resistance, and metastasis [14]. Recent studies have revealed that HSP27 enhances invasion and migration in breast cancer cells, mediates EMT in lung cancer and prostate cancer cells and has been implicated as an inducer of EMT during kidney fibrosis [23–26]. In the present study, it was found that endogenous level of HSP27 reduced with COE concentration. While the expression levels of its mRNA was not changed remarkably. Of interest, we found that the proteasome inhibitor MG132 incubation could restore the HSP27 level following COE treatment. Therefore, COE treatment could probably induce degradation of HSP27 in SGC-7901 cells. Our data also show that overexpression of HSP27 promotes cell invasion and migration and induces EMT process in gastric cancer. These data are consistent with previous studies, suggesting that HSP27 plays an important role in the development of gastric cancer’s metastatic characteristics. Moreover, overexpression of HSP27 weakens the inhibitory effect of COE on EMT, suggesting that inhibition of HSP27 is a primary event in the anti-metastatic activity of COE.

RETRACTED

The NF-κB signaling pathway is involved in the pathogenesis of various cancers, including gastric cancer [27]. Cancer cells in which NF-κB is constitutively active are highly metastatic, and inhibition of NF-κB activity in these cells greatly decreases their invasiveness. The activity of NF-κB is regulated by IκB, which sequesters NF-κB in the cytoplasm, resulting in the inhibition of NF-κB activity. Stimulus-induced phosphorylation and ubiquitination of IκB by the IκB kinase complex have been reported to result in proteasome-mediated degradation, which in turn causes nuclear translocation and DNA binding of NF-κB [28]. In the present study, utilizing western blot and luciferase reporter gene assays, we further confirmed that TNF-α can indeed increase NF-κB transcriptional activity. However, administration of COE can markedly inhibit TNF-α-induced NF-κB transcriptional activity in SGC-7901 cells.

The transcription factor Snail, one of the target genes of NF-κB, is a key regulatory factor in EMT. Snail transcriptionally suppresses the adherent junction protein, E-cadherin, by binding to E2-box type elements within its promoter, resulting in EMT [29]. In this study, we found that COE has a significant inhibitory effect on Snail expression, which is consistent with the blockade of NF-κB by COE. These results suggest that the mechanism of COE to inhibit EMT process may involve the suppression of TNF-α-induced NF-κB/Snail signal pathway.

Recent evidence highlighted that HSP27 enhances the degradation of ubiquitinated proteins by 26S proteasome. Among these ubiquitinated proteins, phosphorylated IκBα could form a complex with HSP27 and 26S proteasome and HSP27 could enhance NF-κB activity by facilitating proteasome mediated IκBα degradation [30]. It seems likely that regulation of HSP27 on NF-κB/Snail signal pathway is involved in the EMT process. Thus, we aimed to clarify whether HSP27 was involved in the action of COE-regulated NF-κB/Snail signal pathway in SGC-7901 cells. In the study, it was found that the overexpression of HSP27 decreased the inhibitory effect of COE on the nuclear translocation of NF-κB p65 and Snail, as well as the phosphorylation of IκBα. It is indicated that HSP27 played a critical role in the process of COE-inhibited NF-κB/Snail signal pathway and offer a new perspective on the role of COE in preventing the procession of cancer.

Peritoneal metastasis is the most common type of metastasis in advanced gastric cancer, and it has a strong negative effect on prognosis of patients [31]. Recent reports have shown a close relation between EMT and peritoneal metastasis in gastric cancer [32, 33]. In the present study, we investigated the role of COE on the peritoneal dissemination in nude mice models. Our results show that COE significantly inhibits the peritoneal dissemination and the expression of HSP27 *in vivo*, which provides a scientific proof to treat patients with gastric cancer by the rationale in the research. Although previous studies suggest that HSP27 possesses different functions, the roles of HSP27 in peritoneal dissemination and in regulating EMT progression remain poorly understood. The present study showed that HSP27 inhibition by COE markedly diminished tumor peritoneal dissemination in a nude mice model. These changes are consistent with the results *in vitro*. Therefore, inhibition of HSP27 may offer new targets for therapeutic intervention to suppress EMT and cancer metastasis.

RETRACTED

In the study, it demonstrated that COE had a satisfactory anti-tumor activity through inhibition of the TGF-β1 induced EMT process in human gastric cancer cell line and had a potent anti-metastasis effect in the peritoneal metastasis model. Thus, COE may become the potential therapy against metastasis. Further studies are needed to identify the metabolism and pharmacokinetics in animal models. In addition, we also need to confirm whether COE and the molecular mechanism identified in the present study had the function in other tumor types.

## Conclusion

Taken together, the present study discovered that COE is a potential inhibitor of HSP27 in human gastric cancer. COE inhibited the EMT by suppressing the expression of HSP27, correlating with inhibition of NF-κB/Snail signal pathway. These data combined with animal model strongly supported COE to be a novel anti-cancer drug candidate, especially for the cancer with abnormal high expression of HSP27. These findings reveal that application of COE in treating metastatic gastric cancer boasts promising prospect and will become potential therapy all over the world.
